The article "Liraglutide Effect on Weight, Glycated Hemoglobin, and Blood Pressure: A Single-Center Experience in the Eastern Province of Saudi Arabia" was retracted in 2022. Reasons: no approval from an author; concerns about the authorship.

# Liraglutide Effect on Weight, Glycated Hemoglobin, and Blood Pressure: A Single-Center Experience in the Eastern Province of Saudi Arabia

**DOI:** 10.7759/cureus.23554

**Published:** 2022-03-27

**Authors:** Duaa M Alsafwani, Hind N Alotaibi, Jawaher A Alzaid, Amal Alghamdi, Huda M Almakhaita

**Affiliations:** 1 Family and Community Medicine, Imam Abdulrahman Bin Faisal University, Dammam, SAU

**Keywords:** glp-1 analogs, saudi arabia, weight, blood pressure, glycated hemoglobin (hba1c), liraglutide

## Abstract

Background

Liraglutide has pleiotropic effects beneficial to patients with cardiovascular and renal risks. These effects have been linked to weight and blood pressure reduction in type 2 diabetes (T2D) patients. However, whether this reduction is similar in all patients regardless of their ethnicity, baseline demographic, or clinical characteristics is unknown. This study aimed to identify the efficacy of liraglutide on weight, glycated hemoglobin (HbA1c), and blood pressure in Saudi patients with T2D who attended King Fahad Hospital of the University and received liraglutide as add-on therapy to other antihyperglycemic agents. The study also aimed to describe the pattern of change in these clinical parameters before and after the treatment and assess whether sex differences affect liraglutide's efficacy.

Methods

We conducted a retrospective longitudinal study reviewing medical records of 220 Saudi patients with T2D treated at King Fahad Hospital of the University (KFHU), in Al-Khobar city in the Eastern Province of Saudi Arabia, from December 2016 to November 2021. Patient cases were included if the patient was Saudi, aged 18 or older, and received liraglutide in a dose of at least 0.6 mg/day for at least three months in combination with other antihyperglycemic agents/diabetes medications. We recorded the effect on patient HbA1c, systolic blood pressure (SBP) and diastolic blood pressure (DBP), body mass index (BMI), and body weight at baseline, during, and after treatment. We used the paired t-test and repeated measure analysis of variance to compare the mean study parameters before and after treatment. Furthermore, an independent t-test was used to compare the mean study parameters among men and women.

Results

Treatment with liraglutide from 0.6 mg/day to 3 mg/day for three to 18 months had optimal results across the outcomes measured in our cohort study. There was a significant reduction in weight from baseline to 18 months from a mean weight of 97.9±20 kg to 96.51±18.45 kg with (p<0.001). Mean HbA1c at baseline was 9.34%±1.95%, dropped to 7.67%±1.11% (p<0.001) at 18 months. Moreover, mean SBP also significantly decreased from 126.61±10.4 mmHg to 122.48±7.29 mmHg by the last follow-up (p<0.001). Mean DBP was 76.54±8.37 mmHg at baseline and decreased to 74.29±6.22 mmHg at last follow-up (p<0.001). Men treated with liraglutide had greater reductions in weight than women throughout the study (p<0.05), and while men had greater reductions in SBP and DBP than women early in treatment (p<0.05), by the end of treatment, there were no significant differences in blood pressure between men and women. Likewise, we saw no significant difference between HbA1c reductions in men and women treated with liraglutide.

The article "Liraglutide Effect on Weight, Glycated Hemoglobin, and Blood Pressure: A Single-Center Experience in the Eastern Province of Saudi Arabia" was retracted in 2022. Reasons: no approval from an author; concerns about the authorship.

Conclusion

Liraglutide effectively reduces HbA1c, weight, BMI, SBP, and DBP in T2D patients. These study results reflect real-world liraglutide clinical practices from KFHU and can be beneficial for physicians when considering using liraglutide as add-on therapy in this population.

## Introduction

Liraglutide is a chemically modified human glucagon-like peptide-1 (GLP-1) receptor agonist. It was approved by the United States Food and Drug Administration in 2010 to boost glycemic control in adult patients with type 2 diabetes (T2D). In 2015, it was approved in higher doses than those used in T2D management for treating obesity and high body mass index (BMI) in patients with a BMI≥30 kg/m^2 ^or those with a BMI≥27 kg/m^2^ with at least one weight-related comorbid condition, such as high blood pressure, T2D, or dyslipidemia [1]. This approval was followed by the Saudi Food and Drug Authority approval in 2016 for the same indications.

Both medically approved versions of liraglutide are instrumental in reducing the risk of cardiovascular factors, including high blood glucose, overweight and obesity issues, high blood pressure, and other severe heart complications like stroke and heart attacks in adults [2-4]. Liraglutide is a once-daily noninsulin medicine essential for lowering glycated hemoglobin (HbA1c) levels and other cardiovascular risk factors [3-6].

The approval of liraglutide was a significant medical breakthrough considering that the risk of cardiovascular complications is the primary cause of death and morbidity globally [7,8]. Estimates from a report by the International Diabetes Federation indicated that by 2035, 59.2 million patients would have diabetes [9]. According to the World Health Organization, 32% of all global deaths in 2019 resulted from cardiovascular complications (17.9 million deaths) [10]. Most of these deaths (85%) involved stroke or heart attack [10].

Obesity is widespread across the Kingdom of Saudi Arabia (KSA), and it increases the likelihood of hypertension, certain types of cancer, osteoarthritis, cardiovascular disease, various non-communicable diseases, and T2D [8]. These diseases lower people's productivity and significantly burden the healthcare system worldwide. Although the prevalence of obesity has been rising globally, the increase is greater in KSA than in many other nations. The estimated incidence in KSA is 35.4%, which is higher than that of nearby Sudan, Syria, Oman, Iraq, and the United Arab Emirates, where the prevalence rates are 8.6%, 27.8%, 27%, 30.4%, and 31.7%, respectively [11].

The article "Liraglutide Effect on Weight, Glycated Hemoglobin, and Blood Pressure: A Single-Center Experience in the Eastern Province of Saudi Arabia" was retracted in 2022. Reasons: no approval from an author; concerns about the authorship.

For people with diabetes and obesity, modest weight loss is important. When people with T2D lose weight, their body's glucose tolerance can improve, allowing them to utilize insulin better [12]. Moreover, losing weight helps protect people with T2D from developing heart disease, liver damage, stroke, hypertension, kidney failure, neuropathy, retinopathy/eye diseases, and other diabetes-related complications [13]. Therefore, there has been a growing interest in medications that can effectively support weight reduction and reduce cardiovascular risk factors. The primary goal of our study was to identify the efficacy of liraglutide on weight, HbA1c, and blood pressure in Saudi patients with T2D who attended King Fahad Hospital of the University (KFUH) and received liraglutide as add-on therapy to other antihyperglycemic agents.

## Materials and methods

We conducted a retrospective longitudinal review of the medical records of 220 patients treated at KFUH in Al-Khobar city in the Eastern Province of Saudi Arabia from December 2016 to November 2021. The study included Saudi 18 years or older patients with T2D who received liraglutide in a dose of at least 0.6 mg/day for at least three months. Patients were excluded from the study if they were non-Saudis, received liraglutide in a dose <0.6mg/day for less than three months, had bariatric surgery during the treatment course or were diagnosed with thyroid disorders, iron deficiency anemia, or hypertension treated with medication. Figure 1 presents the flow chart for patient inclusion and classification.

**Figure 1:** The flow chart for patient inclusion and classification KFUH - King Fahad Hospital of the University

Sample size

The minimal sample size required to represent the whole population was calculated using Epi Info™ for mobile software (US Centers for Disease Control and Prevention, Atlanta, GA). The calculation included the total number of patients treated at KFUH and received liraglutide (n=359), the prevalence of weight reduction was assumed to be 50%, the confidence interval was assumed to be 95%, the margin of error was assigned to be 4.1%, the design effect was 1.0, and the cluster was 1.

Data collection techniques and tools

We reviewed relevant electronic health records (EHRs) at KFUH for patients receiving liraglutide during the study. We documented patient sex, sociodemographic data, use of liraglutide (doses and duration), weight before and after liraglutide use, height, HbA1c, systolic blood pressure (SBP), diastolic blood pressure (DBP), comorbidities, history of bariatric surgery, lifestyle, diet, smoking status, and use of other medications. Patient records that met the inclusion criteria were imported to a Microsoft Excel (Microsoft, Redmond, USA) spreadsheet, then transferred to IBM SPSS Statistics for Windows, Version 28.0. (IBM Inc., Armonk, USA) for analysis.

The article "Liraglutide Effect on Weight, Glycated Hemoglobin, and Blood Pressure: A Single-Center Experience in the Eastern Province of Saudi Arabia" was retracted in 2022. Reasons: no approval from an author; concerns about the authorship.

Data processing and analysis

Frequency tables were drawn to explore the findings. Measures of central tendency and measures of dispersion were calculated for quantitative data. We used frequency and percentage tables for categorical variables' descriptions to assess relationships. We used paired t-test and repeated measure analysis of variance to compare the mean study parameters before and after treatment. Furthermore, an independent t-test was used to compare the mean study parameters among men and women. We considered p<0.05 as statistically significant.

A pilot study performed on a random sample of 10 EHR cases confirmed the feasibility and accessibility of the main study design. A reliability test was conducted using Cronbach's Alpha test (Table 1). If the Alpha value is >0.70, the data are considered reliable. Since Cronbach's Alpha was 0.921, the data are considered reliable.

**Table 1:** Reliability statistics

Cronbach's Alpha	Cronbach's Alpha based on standardized items	N of items
0.921	0.852	36

Ethical considerations

Before the study began, we received approval from the relevant Institutional Review Board (IRB-PGS-2020-01-419). We maintained patient confidentiality, and no identifying information was collected or divulged.

## Results

Two hundred twenty cases were included in the study. The mean age of the study population was 51.2±12.4 years; the mean weight was 97.9±20 kg, mean BMI was 36.45±7.58 kg/m^2^, mean HbA1c was 9.34%±1.95%, mean SBP was 126.6±10.4 mmHg, and the mean DBP was 76.5±8.3 mmHg. The study population consisted of 131 women (59.5%) and 89 men (40.5%). Most participants were married (n=167, 76.3%) and unemployed (n=159, 72.3%; see Table 2).

**Table 2:** Sociodemographic and baseline characteristics of the participants NA - not applicable; BMI - body mass index; SD - standard deviation; HbA1c - glycated hemoglobin; SBP - systolic blood pressure; DBP - diastolic blood pressure

Variables	N (%)	Mean ± SD (range)
Sex		
Male	89 (40.5%)	NA
Female	131 (59.5%)	NA
Total	220 (100%)	NA
Marital status		
Single	48 (21.9%)	NA
Married	167 (76.9%)	NA
Divorced	2 (0.9%)	NA
Widowed	3 (1.4%)	NA
Total	220 (100%)	NA
City of residence		
Al-Ahsa	5 (2.3%)	NA
Dhahran	18 (8.2%)	NA
Dammam	55 (25%)	NA
Khobar	111 (50.5%)	NA
Qatif	14 (6.4%)	NA
Other	17 (7.7%)	NA
Total	220 (10%)	NA
Occupational status		
Employed	61 (27.7%)	NA
Unemployed	159 (72.3%)	NA
Total	220 (100%)	NA
Nationality		
Saudi	220 (100%)	NA
Non-Saudi	0 (0%)	NA
Total	220 (100%)	NA
Age in years	NA	51.2±12.4 (20 - 81)
Weight in Kg	NA	97.9±20 (59 - 164)
Height in cm	NA	164.21±9.75 (142 - 190)
BMI in kg/m^2^	NA	36.45±7.58 (22.04 - 71.62)
HbA1c in percentage	NA	9.34±1.95 (5 - 16)
SBP in mmHg	NA	126.6±10.4 (100 - 156)
DBP in mmHg	NA	76.5±8.3 (53 - 96)

Table 3 presents the baseline medical and surgical history. Over half of the population (n=127, 57.7%) were on a calorie-restricted diet, 46.8% of patients (n=103) reported exercising, and only nine received bariatric surgery before (n=5) or after (n=4) the study period. All patients had T2D (100%), 112 had coronary artery disease (50.9%), 110 had dyslipidemia (50%), and four patients had a stroke or transient ischemic attack (1.8%).

The article "Liraglutide Effect on Weight, Glycated Hemoglobin, and Blood Pressure: A Single-Center Experience in the Eastern Province of Saudi Arabia" was retracted in 2022. Reasons: no approval from an author; concerns about the authorship.

**Table 3:** Baseline medical and surgical history of the participants DVT - deep vein thrombosis; PE - pulmonary embolism; COPD - chronic obstructive pulmonary disease; T2D - type 2 diabetes; PCOS - polycystic ovary syndrome; TIA - transient ischemic attack

Variables	Yes, n (%)	No, n (%)
Calorie-restricted diet	127 (57.7%)	93 (42.3%)
Exercise	103 (46.8%)	117 (53.2%)
Smoking	30 (13.6%)	190 (86.4%)
Bariatric surgery was done before the treatment course	5 (2.3%)	215 (97.72%)
Bariatric surgery was done after the treatment course	4 (1.8%)	216 (98.18%)
Coronary artery disease	112 (50.9%)	108 (49.1%)
Peripheral artery disease	2 (0.9%)	218 (99.1%)
Stroke/TIA	4 (1.8%)	216 (98.2%)
DVT/PE	3 (1.4%)	217 (98.6%)
T2D	220 (100%)	0 (0.0%)
Dyslipidemia	110 (50%)	110 (50%)
Bronchial asthma	19 (8.6%)	201 (91.4%)
COPD	4 (1.8%)	216 (98.2%)
Obstructive sleep apnea	12 (5.5%)	208 (94.5%)
Obesity hypoventilation syndrome	1 (0.5%)	219 (99.5%)
Chronic kidney disease / end-stage renal disease	8 (3.6%)	218 (99.1%)
Gallbladder disease (cholecystitis, cholelithiasis)	2 (0.9%)	218 (99.1%)
Nonalcoholic fatty liver disease	4 (1.8%)	216 (98.2%)
Osteoarthritis	6 (2.7%)	214 (97.3%)
Chronic back pain / chronic lumbago	6 (2.7%)	214 (97.3)
PCOS	3 (1.4%)	217 (98.6%)
Infertility	9 (4.1%)	211 (95.9%)
Depression	13 (5.9%)	207 (94.1%)

Table 4 presents the different liraglutide doses over the follow-up period. At the beginning of the study, most patients (n=191, 86%) received 0.6 mg/day of liraglutide. Throughout the follow-up period, a majority received 1.8 mg/day (76.4% at three months), then the proportion of patients receiving this dose declined over time (68.6% at six months, 61.4% at nine months, 51.4% at 12 months, and 41.4% at 18 months).

The article "Liraglutide Effect on Weight, Glycated Hemoglobin, and Blood Pressure: A Single-Center Experience in the Eastern Province of Saudi Arabia" was retracted in 2022. Reasons: no approval from an author; concerns about the authorship.

**Table 4:** Liraglutide doses over the follow-up period

Dose	At 0 months, n (%)	At 3 months, n (%)	At 6 months, n (%)	At 9 months, n (%)	At 12 months, n (%)	At 18 months, n (%)
0.6 mg	191 (86.8%)	17 (7.7 %)	11 (5.0%)	5 (2.3%)	2 (0.9%)	0 (0%)
1.2 mg	22 (10%)	27 (12.3%)	6 (2.7%)	2 (0.9%)	2 (0.9%)	2 (0.9%)
1.8 mg	7 (3.2%)	168(76.4%)	151 (68.6%)	135 (61.4%)	113 (51.4%)	99 (41.4%)
2.4 mg	0 (0%)	2 (0.9 %)	1 (0.5%)	3 (1.4%)	5 (2.3%)	2 (0.9%)
3 mg	0 (0%)	6 (2.7%)	4 (1.8%)	4 (1.8%)	4 (1.8%)	3 (1.4%)
Total	220	220	173	149	126	99

Table 5 presents participants' baseline medications. Patients received a variety of antihyperglycemic medications. All participants received liraglutide, 187 patients (85%) received metformin, 154 patients (70%) received insulin, 121 patients (55%) received sodium-glucose cotransporter-2 inhibitors, 52 (23.6%) received sulfonylurea, and no patients received dipeptidyl peptidase-4 inhibitors or alpha-glucosidase inhibitors. Forty-nine patients (22.3%) received steroids.

**Table 5:** Baseline medication of the participants DPP-4 - dipeptidyl peptidase-4; GLP-1 RA - glucagon-like peptide-1 receptor agonist; SGLT-2 - sodium-glucose cotransporter-2; TZD - thiazolidinedione

Medication	N (%)
Antihyperglycemic / diabetes medication	
Metformin	187 (85%)
Insulin	154 (70%)
DPP-4	0 (0%)
GLP-1 RA inhibitor	220 (100%)
SGLT-2 inhibitor	121 (55%)
Sulfonylurea	52 (23.6%)
Alpha-glucosidase inhibitor	0 (0%)
Antidepressants and anxiolytics	14 (6.4%)
Antipsychotics	4 (1.8%)
Anticonvulsants	17 (7.7%)
Opioids	2 (0.9%)
Steroid	49 (22.3%)
TZD	17 (7.7%)

The frequency and percentage of patient follow-up sessions are presented in Table 6. While the initial population was 220 patients, only 173 had data available (78.6%) at six months; 149 remained (67.7%) at nine months. After 12 months of follow-up, data from 125 patients remained (56.8%), and at 18 months, data from 98 patients were available (44.5%). 

**Table 6:** Participants according to the duration of the liraglutide treatment course

Duration of the liraglutide treatment course	N (%)
At 0 months	220 (100%)
At 3 months	220 (100%)
At 6 months	173 (78.6%)
At 9 months	149 (67.7%)
At 12 months	126 (56.8%)
At 18 months	99 (44.5%)

We recorded changes over time in clinical parameters, including weight, BMI, HbA1c, SBP, and DBP in Table 7, and Table 8 presents the pretreatment and posttreatment statistical analyses. At the three-month follow-up, the mean weight decreased from 97.9±20 kg to 95±19.88 kg (p<0.001). As of the last follow-up, mean BMI also significantly decreased from 36.45±7.58 kg/m^2^ to 35.02±7.42 kg/m^2^ (p<0.001). We noted a significant decrease in mean HbA1c from 9.34%±1.95% at baseline to 7.67%±1.11% at the last follow-up (p<0.001). Mean SBP also significantly decreased from 126.61±10.4 mmHg to 122.48±7.29 mmHg by the last follow-up (p<0.001). Mean DBP was 76.54±8.37 mmHg at baseline and decreased to 74.29±6.22 mmHg at the last follow-up (p<0.001).

The article "Liraglutide Effect on Weight, Glycated Hemoglobin, and Blood Pressure: A Single-Center Experience in the Eastern Province of Saudi Arabia" was retracted in 2022. Reasons: no approval from an author; concerns about the authorship.

**Table 7:** Changes in mean clinical parameters over time SD - standard deviation; BMI - body mass index; NA - not applicable; HbA1c - glycated hemoglobin; SBP - systolic blood pressure; DBP - diastolic blood pressure

Variables	At 0 months	At 3 months	At 6 months	At 9 months	At 12 months	At 18 months / at the end of the course	p-value
Mean weight ± SD (range)	97.9±20 kg (59 - 164 kg)	95.53±19.88 kg (57 - 160 kg)	95.54±19.32 kg (52 - 159 kg)	95.26±19.57 kg (52 - 157 kg)	96.41±19.58 kg (63 - 157 kg)	96.51±18.45 kg (63 - 157 kg)	<0.001
Total	220	220	173	149	126	99	
Mean BMI ± SD (range)	36.45±7.58 kg/m^2 ^(22.04 - 71.62 kg/m^2^)	NA	NA	NA	NA	35.02±7.42 kg/m^2^ (23.31 - 70.27 kg/m^2^)	<0.001
Total	220					220	
Mean HbA1c ± SD (range)	9.34±1.95 (5 - 16)	8.44±1.66 (4.9 - 13.7)	8.16±1.45 (5.1 - 13)	8.02±1.34 (5.3 - 11.7)	7.84±1.18 (5.3 - 11.6)	7.675±1.11 (4.9 - 10.5)	<0.001
Total	220	220	173	149	126	99	
Mean SBP ± SD (range)	126.61±10.4 mmHg (100 - 156 mmHg)	123.7±8.35 mmHg (105 - 156 mmHg)	123.32±8.35 mmHg (100 - 163 mmHg)	122.27±7.86 mmHg (100 - 145 mmHg)	122.66±7.88 mmHg (106 - 149 mmHg)	122.48±7.29 mmHg (106 - 139 mmHg)	<0.001
Total	220	220	173	149	126	99	
Mean DBP ± SD (range)	76.54±8.37 mmHg (53 - 96 mmHg)	74.6±6.91 mmHg (57- 90 mmHg)	74.56±7.2 mmHg (59 - 92 mmHg)	73.1±6.46 mmHg (51 - 86 mmHg)	74.06±6.84 mmHg (54 - 93 mmHg)	74.29±6.22 mmHg (57 - 88 mmHg)	<0.001
Total	220	220	173	149	126	99	

**Table 8:** Difference between pretreatment and posttreatment clinical parameters SD - standard deviation; BMI - body mass index; HbA1c - glycated hemoglobin; SBP - systolic blood pressure; DBP - diastolic blood pressure

Pre difference to post difference	Mean difference	SD	95% confidence interval of the difference		t-value	p-value
			Lower	Upper		
Weight at 0 & 3 months	2.377	1.818	2.136	2.619	19.397	<0.001
Weight at 0 & 6 months	3.610	2.033	3.304	3.916	23.289	<0.001
Weight at 0 & 9 months	4.014	1.945	3.698	4.329	25.107	<0.001
Weight at 0 & 12 months	4.183	2.033	3.824	4.541	23.090	<0.001
Weight at 0 & 18 months	4.290	2.157	3.862	4.718	19.889	<0.001
BMI at 0 months and at the end of the course	1.427	0.877	1.31	1.543	24.117	<0.001
HbA1c at 0 & 3 months	0.895	0.802	0.788	1.001	16.549	<0.001
HbA1c at 0 & 6 months	1.254	0.937	1.113	1.394	17.608	<0.001
HbA1c at 0 & 9 months	1.404	0.979	1.245	1.562	17.497	<0.001
HbA1c at 0 & 12 months	1.566	1.094	1.373	1.759	16.075	<0.001
HbA1c at 0 & 18 months	1.688	1.136	1.462	1.915	14.780	<0.001
SBP at 0 & 3 months	2.909	5.964	2.116	3.701	7.234	<0.001
SBP at 0 & 6 months	4.271	8.461	3.001	5.541	6.640	<0.001
SBP at 0 & 9 months	5.288	8.373	3.933	6.644	7.710	<0.001
SBP at 0 & 12 months	5.253	8.625	3.733	6.774	6.837	<0.001
SBP at 0 & 18 months	5.707	8.626	3.986	7.427	6.583	<0.001
DBP at 0 & 3 months	1.940	6.206	1.116	2.765	4.638	<0.001
DBP at 0 & 6 months	2.491	8.318	1.243	3.739	3.939	<0.001
DBP at 0 & 9 months	4.160	8.282	2.823	5.496	6.151	<0.001
DBP at 0 & 12 months	3.357	7.705	1.998	4.715	4.891	<0.001
DBP at 0 & 18 months	3.444	7.443	1.959	4.929	4.604	<0.001

The differences in liraglutide effects on clinical parameters, weight, HbA1c, SBP, and DBP according to patient sex are presented in Table 9. Liraglutide had a significantly greater effect on weight at time of treatment (p=0.009), three (p=0.008), six (p=0.007), nine (p=0.004), 12 (p=0.003), and 18 months (p=0.020). Liraglutide had a more significant effect on SBP reduction in men than women at the time of treatment (p=0.009) and three months (p=0.008), but no significant differences were seen between men and women at six (p=0.804), nine (p=0.308), 12 (p=0.191), and 18 months (p=0.065). Liraglutide treatment in men also had a significantly greater effect on DBP than women at the time of treatment (p=0.02), three (p=0.02), nine (p=0.032), and 12 months (p=0.036). There were no statistically significant differences in DBP between men and women six months (p=0.713) and 18 months (p=0.111). Throughout the study, we found no statistically significant differences in changes to HbA1c between men and women treated with liraglutide.

The article "Liraglutide Effect on Weight, Glycated Hemoglobin, and Blood Pressure: A Single-Center Experience in the Eastern Province of Saudi Arabia" was retracted in 2022. Reasons: no approval from an author; concerns about the authorship.

**Table 9:** Comparison of clinical parameters by sex BMI - body mass index; HbA1c - glycated hemoglobin; SBP - systolic blood pressure; DBP - diastolic blood pressure

Variable	Male	Female	Mean difference	p-value
Weight at 0 months	102.13±20.464	95.03±19.21	7.104	0.009
	(n=89)	(n=131)		
Weight at 3 months	99.85±20.547	92.59±18.93	7.266	0.008
	(n=89)	(n=131)		
Weight at 6 months	100.24±20.58	92.24±17.75	8.002	0.007
	(n=71)	(n=102)		
Weight at 9 months	100.71±21.10	91.34±17.47	9.372	0.004
	(n=62)	(n=87)		
Weight at 12 months	102.31±21.42	91.99±16.907	10.329	0.003
	(n=54)	(n=72)		
Weight at 18 months	100.76±18.72	91.27±18.88	8.500	0.020
	(n=50)	(n=49)		
HbA1C at 0 months	9.21±2	9.41±1.91	-0.166	0.537
	(n=89)	(n=131)		
HbA1C at 3 months	8.31±1.62	8.53±1.68	-0.2175	0.341
	(n=89)	(n=131)		
HbA1C at 6 months	8.07±1.40	8.22±1.488	-0.146	0.516
	(n=71)	(n=102)		
HbA1c at 9 months	7.79±1.32	8.17±133	-0.375	0.091
	(n=62)	(n=87)		
HbA1c at 12 months	7.62±1.17	7.99±1.77	-0.376	0.077
	(n=54)	(n=72)		
HbA1c at 18 months	7.61±1.24	7.87±1.44	-0.320	0.154
	(n=50)	(n=49)		
SBP at 0 months	128.81±10.29	125.11±10.25	3.69	0.009
	(n=89)	(n=131)		
SBP at 3 months	125.52±8.488	122.47±8.05	3.05	0.008
	(n=89)	(n=131)		
SBP at 6 months	123.51±7.98	123.19±8.63	0.32	0.804
	(n=71)	(n=102)		
SBP at 9 months	123.04±8.19	121.71±7.60	1.33	0.308
	(n=62)	(n=87)		
SBP at 12 months	123.72±8.5	121.86±7.27	1.86	0.191
	(n=54)	(n=72)		
SBP at 18 months	123.82±7.09	121.12±7.31	2.69	0.065
	(n=50)	(n=49)		
DBP at 0 months	78.12±8.35	75.47±8.24	2.65	0.020
	(n=89)	(n=131)		
DBP at 3 months	75.84±6.55	73.76±7.05	2.08	0.020
	(n=89)	(n=131)		
DBP at 6 months	74.80±6.17	74.39±7.86	0.41	0.713
	(n=71)	(n=102)		
DBP at 9 months	74.41±5.93	72.17±6.68	2.24	0.032
	(n=62)	(n=87)		
DBP at 12 months	75.53±7.2	72.95±6.37	2.57	0.036
	(n=54)	(n=72)		
DBP at 18 months	75.28±6.11	73.29±6.22	1.99	0.111
	(n=50)	(n=49)		

## Discussion

This study aimed to identify the efficacy of liraglutide on weight, HbA1c, and blood pressure in Saudi patients with T2D who attended KFUH and received liraglutide as add-on therapy to other antihyperglycemic agents. While similar studies have been conducted on other ethnic populations [14,15], this study is the first such study conducted in a Saudi population.

Most of the 220 patients included in our study were women (59.5%), which aligns with previous reports that T2D is more common in female patients [16], including those by Pi-Sunyer et al. (78.7%) [17] and Fujishima et al. (59%) [14]. Most patients in the study were overweight, with a mean BMI of 36.45±7.58 kg/m^2^, and given that obesity is highly associated with T2D, this finding is not surprising [18]. The high mean HbA1c, SBP, and DBP among study participants indicate poor diabetic control and evidence of elevated blood pressure. Moreover, many patients had dyslipidemia (50%) and coronary artery disease (50.9%). These concurrent characteristics among our participants indicate they were appropriate candidates for the study.

Weight reduction has a significant impact on the cardiovascular outcomes of patients with diabetes [18]. Sanjoy et al. reported that cardiovascular outcomes significantly improved in patients with T2D who received exenatide (a GLP-1 receptor agonist) or exenatide plus insulin compared to those receiving insulin only [19]. Likewise, it is expected that liraglutide can enhance cardiovascular outcomes in patients with T2D, given the significant reduction of weight associated with liraglutide treatment demonstrated in our study. We saw a significant reduction in mean weight from 97.9±20 kg at the beginning of the study to 96.51±18.45 kg at the end of the study (p<0.001). This finding is consistent with a cohort study on Arabian people with T2D who received liraglutide, where weight loss ranged between 0.5 and 17 kg and the mean weight loss was 2.5±0.6 kg [20]. In addition, the Liraglutide Effect and Action in Diabetes (LEAD) study reported weight loss of 1.8 to 3.2 kg, depending on the dose of liraglutide and the combination therapy used in the program [21]. However, contrary to our findings, Kendall et al.'s meta-analysis on incretin-based therapies in the Asian population with T2D concluded that of all GLP-1 receptor agonist analogs, exenatide was the only drug that resulted in significant weight loss in an Asian population. At the same time, liraglutide was weight neutral [22]. This difference may be attributed to different ethnic groups in both studies.

The article "Liraglutide Effect on Weight, Glycated Hemoglobin, and Blood Pressure: A Single-Center Experience in the Eastern Province of Saudi Arabia" was retracted in 2022. Reasons: no approval from an author; concerns about the authorship.

Previous studies have reported that liraglutide is effective in helping to control hyperlipidemia, with a reduction in total cholesterol of 5.01 mg/dl from baseline after liraglutide treatment [23]. While our study did not assess dyslipidemia, it is reasonable to expect a positive effect on dyslipidemia secondary to the observed improvement of weight, HbA1c, and blood pressure.

Liraglutide effectively reduces HbA1c as monotherapy and in combination with oral antihyperglycemic agents, as demonstrated in the LEAD 2 and LEAD 3 studies [24,25]. Treatment with liraglutide resulted in 1.2% to 1.6% reduction in HbA1c at 1.2 to 1.8 mg doses. In LEAD 5, a larger percentage of patients achieved an HbA1c <7 % and <6.5 % with liraglutide than those on metformin, glimepiride, and glargine [22]. We noted a significant decrease in mean HbA1c from 9.34%±1.95% at baseline to 7.67%±1.11% at the last follow-up (p<0.001). These results are consistent with those from a cohort study on an Arabic population that demonstrated a significant reduction in HbA1c that ranged from 0.5% to 1.15% in six months [20]. Moreover, Mirabelli et al. reported that HbA1c decreased from 7.9%±0.9% at baseline to 7.0%±0.7% at the end of their study period (p<0.001), along with a significant reduction in fasting plasma glucose in diabetic patients treated with liraglutide as a combination therapy [26].

Mean SBP and DBP significantly decreased in our study, which was likely due to the positive effects of weight and diabetes control on blood pressure or the direct antihypertensive effect of liraglutide. This supports findings reported by Robinson et al. in their meta-analysis, who noted that GLP-1 receptor agonists significantly decreased SBP in patients with T2D compared to placebo and active controls [27]. However, the reduction in DBP was not significant in their analysis. Zhao et al. also conducted a meta-analysis on the effect of liraglutide on systemic blood pressure using 18 randomized controlled trials that enrolled 7,616 individuals in the liraglutide group and 6,046 in the control group [28]. Compared with placebo, liraglutide reduced SBP by 3.18 mmHg (95% confidence interval [CI], 4.32 to 2.05; p<0.0001), but it had no significant effect on DBP. Zhao et al. also conducted a dose-dependent subgrouping and analysis and found that the degree of reduction in SBP was associated with the dose of liraglutide, but that significance disappeared when the intervention lasted over one year [28]. In their analysis, a liraglutide dose of 3.0 mg/day significantly reduced DBP by 1.46 mmHg (95% CI, 2.61 to 0.32). Therefore, SBP reduction in patients with T2D using liraglutide is not dose-dependent during long-term treatment. It also indicates that a dose-dependent DBP reduction was observed and that further studies might be required to confirm this finding.

The article "Liraglutide Effect on Weight, Glycated Hemoglobin, and Blood Pressure: A Single-Center Experience in the Eastern Province of Saudi Arabia" was retracted in 2022. Reasons: no approval from an author; concerns about the authorship.

Finally, liraglutide had a significantly greater effect on weight (p=0.003) in men than women. Liraglutide affected SBP and DBP differently in men and women; however, no significant difference in efficacy between the sexes was seen at the end of the study period. This finding of a difference in weight reduction between men and women using liraglutide has not been previously reported and needs further exploring in future studies.

Limitations and strengths of the study

Our study had several important limitations. This was an observational study, which results less solid than those from randomized controlled studies; however, it does not impact its reliability. This study targeted a small part of the Saudi population, limiting our results' generalizability. However, it is the only study thus far to report on the use of liraglutide in the Saudi population and reflects real-world clinical practice in this region. Another limitation of this study is the loss of follow-up for some patients, which reduced the sample size. This study was not designed to look at the safety and tolerability of liraglutide, two facets that would have added value to the study.

## Conclusions

This study aimed to elucidate the effect of liraglutide therapy as an add-on to other antihyperglycemic agents on weight, blood pressure, and diabetic control in patients with T2D. Liraglutide as an add-on therapy is significantly effective in reducing weight, HbA1c, and blood pressure in Saudi patients with T2D. Moreover, liraglutide has a significantly larger weight reduction effect in men than women. Our results provide further insight into the benefits of liraglutide in this part of the world, a medication that might eventually improve the overall health of T2D patients and enhance their cardiovascular outcomes.
